The article "Metal-based 2,3-indolinedione derivatives as proteasome inhibitors and inducers of apoptosis in human cancer cells" was published in 2014. Journal: Int J Mol Med.

# Metal-based 2,3-indolinedione derivatives as proteasome inhibitors and inducers of apoptosis in human cancer cells

**DOI:** 10.3892/ijmm.2014.1838

**Published:** 2014-07-08

**Authors:** PENGFEI ZHANG, CAIFENG BI, SARA M. SCHMITT, XIN LI, YUHUA FAN, NAN ZHANG, Q. PING DOU

**Affiliations:** 1 Key Laboratory of Marine Chemistry Theory and Technology, Ministry of Education, College of Chemistry and Chemical Engineering, Ocean University of China, Qingdao, Shandong 266100, P.R. China; 2 Barbara Ann Karmanos Cancer Institute, Departments of Oncology, Pharmacology and Pathology, School of Medicine, Wayne State University, Detroit, MI 48201, USA

**Keywords:** ubiquitin-proteasome system, metal-based complexes, 2,3-indolinedione derivative, inhibitor, electron-attracting group

## Abstract

Proliferation and apoptotic pathways are tightly regulated in cells by the ubiquitin-proteasome system (UPS). Alterations in the UPS may result in cellular transformation or other pathological conditions. The proteasome is indeed often found to be overactive in cancer cells. It has been reported that 2,3-indolinedione (L), which exists in marine organisms, as well as in mammals, is a proteasome inhibitor. Studies have shown that metal-based complexes inhibit proteasome activity and induce apoptosis in certain human cancer cells. In the current study, we synthesized six novel metal-based complexes with derivatives of 2,3-indolinedione: [Cd (C_15_H_11_O_3_N_2_) (CH_3_COO)] (C1), [Cd (C_15_H_11_O_2_N_2_) (CH_3_COO)] (C2), [Co (C_15_H_9_O_4_N_2_) (CH_3_COO)] (C3), [Co (C_15_H_11_O_2_N_2_) (CH_3_COO)] (C4), [Zn (C_19_H_14_O_3_N_3_) (CH_3_COO)] (C5) and [Zn (C_17_H_13_O_3_N_2_) (CH_3_COO)] (C6). We sought to characterize and assess the proteasome inhibitory and anti-proliferative effects of these metal-based complexes in human breast (MDA-MB-231) and prostate (LNCaP and PC-3) cancer cells, in order to determine whether specific structures contribute to the inhibition of tumor proteasome activity and the induction of apoptosis. The results revealed that the complexes, C1, C3 and C5, but not their counterparts, C2, C4 and C6, inhibited the chymotrypsin-like activity of the human cancer cellular 26S proteasome; in addition, these complexes promoted the accumulation of the proteasome target protein, Bax, inhibited cell growth and induced apoptosis in a concentration- and time-dependent manner due to their unique structures. Our data suggest that the study of metal-based complexes, including aromatic ring structures with electron-attracting groups, may be an interesting research direction for the development of anticancer drugs.

## Introduction

The ubiquitin-proteasome system (UPS) is a major pathway for intracellular protein degradation and regulates a number of key cellular processes. Its target proteins include a broad array of regulatory proteins that play important roles in cell cycle progression, cell development and differentiation, DNA damage response and tumorgenesis. This system allows the cells to modulate their protein expression patterns in response to changing physiological conditions and plays a critical role in health and disease (1,2). The UPS has therefore been extensively studied as a novel molecular target for the development of novel drugs in an attempt to restore protein homeostasis, as the ultimate therapeutic strategy (3,4). The proteasome is a massive multicatalytic protease responsible for degrading a large number of cellular proteins. In order to be degraded by the proteasome, these target proteins are first tagged with ubiquitin (Ub), which can then target the substrate protein to the 26S proteasome for destruction. The 20S proteasome, the core of the 26S proteasome complex, has at least three distinct catalytic activities, including chymotrypsin-like activity (cleavage after hydrophobic residues by the β5 subunit). Several studies have shown that the inhibition of the proteasomal chymotrypsin-like activity results in the accumulation of several target proteins and the induction of apoptosis in various types of tumor cells (5,6).

Zinc (Zn) was recognized as a trace element with important roles in various metabolic processes in living organisms almost a century ago. Zinc is the second most abundant transition metal ion in the human body and an essential element for the proper function of many different enzymes and the tight control of gene expression (7–9). Cobalt (Co) is also needed in the body and is an essential trace element found in small amounts in different organs and bones. It is an integral part of vitamin B12, which is vital to the formation of red blood cells (10,11). Additionally, cadmium (Cd) has been shown to affect cell proliferation, differentiation and apoptosis (12). The interest in metal-based anticancer drugs has increased since the development of cisplatin (13–16); however, due to the fact that there are many pitfalls in the use of metal-based anticancer drugs, the search for other metals and ligands that may produce more specific antitumor effects is an ongoing process, in an effort to synthesize and characterize novel potential metal-based antitumor drugs that have less toxicity and higher clinical effectiveness (18–20). Our laboratory has studied a number of novel metal-based drugs, including organic copper-, zinc- and cadmium-based complexes, capable of inhibiting the tumor cell proteasome and thus, proliferation, thereby inducing cancer cell death (3,17,21–23). It has also been reported that cobalt-based complexes effectively inhibit chymotrypsin-like activity in the purified proteasome and PC-3 prostate cancer cells (24).

2,3-Indolinedione (isatin; formula, C_8_H_5_O_2_N), an endogenous indole in marine and mammalian organisms, possesses a wide range of biological activities, including anxiogenic, sedative and anticonvulsant activities, and is a potent antagonist of atrial natriuretic peptide receptors. Studies have shown that 2,3-indolinedione and its derivatives have pro-apoptotic functions in human cancer and mouse neuroblastoma cells (25,26).

Considering the importance of the UPS and the properties of 2,3-indolinedione, we aimed to investigate whether 2,3-indolinedione derivatives have the ability to inhibit proteasome activity, and whether structure is an essential factor affecting antitumor activity. To investigate our hypothesis, we synthesized six novel metal compounds (Table I) with 2,3-indolinedione, 2-amino-5-methoxyphenol (N1), 2-amino-5-methylphenol (N2), 3-hydroxy-4-aminobenzoic acid (N3), L-tryptophane (N4) and L-phenylalanine (N5) with Cd (M1), Zn (M2) and Co (M3), respectively (Table I). The compounds were then tested in human breast cancer metal-based complexes in human breast (MDA-MB-231) cells to determine whether compound structure affects proteasome-inhibitory and apoptosis-inducing abilities.

## Materials and methods

### Materials

Compounds C1-C6 were synthesized by the laboratory at the Ocean University of China, Qingdao, China. 3-(4,5-Dimethylthiazol-2-yl)-2,5-diphenyltetrazolium bromide (MTT), dimethyl sulfoxide (DMSO) and other chemicals were purchased from Sigma-Aldrich (St. Louis, MO, USA). All compounds were dissolved in DMSO at stock concentrations of 80 mM and stored at 4°C. Fetal bovine serum (FBS) was purchased from Aleken Biologicals (Nash, TX, USA). Dulbecco’s modified Eagle’s medium/F12 medium and penicillin/streptomycin were purchased from Invitrogen (Carlsbad, CA, USA). Rabbit polyclonal antibody against human poly(ADP-ribose) polymerase (PARP; H-250), mouse monoclonal antibodies against Ub (P4D1), Bax (B-9), goat polyclonal antibody against β-actin (C-11) and donkey anti-goat secondary antibody were from Santa Cruz Biotechnology, Inc. (Santa Cruz, CA, USA). Goat anti-rabbit and goat anti-mouse secondary antibodies were from Bio-Rad (Hercules, CA, USA).

### Metal complex syntheses

C1, C2, C3, C4, C5 and C6: these compounds were synthesized by the laboratory at the Ocean University of China. The ligand (2 mM) was dissolved in 15 ml of ethanol. M (CH_3_COO)_2_·2H_2_O (2 mM) dissolved in 10 ml of anhydrous ethanol was added dropwise to the above solution with stirring and the mixture was reacted for 4 h at 50°C to yield a precipitate, which was filtered off, to produce the final complexes.

C1: yield, 81%; Anal. Calc. for C1 {%, [Cd (C_15_H_11_O_3_N_2_) (CH_3_COO)], FW=438.71 g·mol^-1^}; C, 46.54; H, 3.22; N, 6.39. Found (%): C, 47.02; H, 3.19; N, 6.56. λmax (nm): 232, 285. IR data (KBr, cm^-1^): 3267.68, υ (-NH-); 1651.35, υ (-C=O); 1618.32, υ (-C=N-); 1590.95, υ_as_ (COO-); 1319.99, υ_s_ (COO-); 1197.76, υ (-OCH_3_); 1108.84, υ (-Ph-OH); 478.89, υ (Cd-O). 1H NMR (DMSO, 600 MHz; s, singlet; d, doublet; t, triplet): δ (ppm) 10.498 (s, 1H, -NH-); 7.497 (s, 1H, -Ph-H); 7.340 (d, 1H, -Ph-H); 7.066 (s, 1H, -Ph-H); 6.726 (s, 1H, -Ph-H); 6.462 (s, 1H, -Ph-H); 6.438 (d, 1H, -Ph-H); 6.306 (s, 1H, -Ph-H); 3.323 (d, 3H, -OCH3); 2.614 (t, 3H, -CH3). Thermogravimetric (TG) analysis, residue 30.22% (calculated 29.27%, CdO). Molar conductivity, Λm (S·cm^2^·mol^-1^): 19.88.

C2: yield, 85%; Anal. Calc. for C2 {%, [Cd (C_15_H_11_O_2_N_2_) (CH_3_COO)], FW=422.72 g·mol^-1^}; C, 48.30; H, 3.34; N, 6.63. Found (%): C, 48.41; H, 3.31; N, 7.01. λmax (nm): 236, 655. IR data (KBr, cm^-1^): 3189.68, υ (-NH-); 1648.35, υ (-C=O); 1610.52, υ (-C=N-); 1580.95, υ_as_ (COO-); 1327.89, υ_s_ (COO-); 1199.56, υ (-Ph-OH); 470.89, υ (Cd-O). 1H NMR (DMSO, 600 MHz; s, singlet; d, doublet; t, triplet): δ (ppm) 10.498 (s, 1H, -NH-); 7.497 (s, 1H, -Ph-H); 7.340 (d, 1H, -Ph-H); 7.066 (s, 1H, -Ph-H); 6.726 (s, 1H, -Ph-H); 6.462 (s, 1H, -Ph-H); 6.438 (d, 1H, -Ph-H); 6.306 (s, 1H, -Ph-H); 2.614 (t, 3H, -CH3); 2.541 (d, 3H, -CH3). TG analysis: residue 31.32% (calculated 30.74%, CdO). Molar conductivity, Λm (S·cm^2^·mol^-1^): 19.60.

C3: yield, 79%; Anal. Calc. for C3 {%, [Co (C_15_H_9_O_4_N_2_) (CH_3_COO)], FW=399.22 g·mol^-1^}; C, 51.15; H, 3.03; N, 7.02. Found (%): C, 52.25; H, 2.96; N, 7.21. λmax (nm): 238, 564. IR data (KBr, cm^-1^): 3215.46, υ (-NH-); 1678.66, υ (-C=O); 1602.19, υ (-C=N-); 1540.99, υ_as_ (COO-); 1321.62, υ_s_ (COO-); 1212.36, υ (-Ph-OH); 477.02, υ (Co-O). 1H NMR (DMSO, 600 MHz; s, singlet; d, doublet; t, triplet): δ (ppm) 11.308 (s, 1H, -COOH); 10.964 (s, 1H, -NH-); 7.584 (d, 1H, -Ph-H); 7.497 (s, 1H, -Ph-H); 7.340 (d, 1H, -Ph-H); 7.065 (s, 1H, -Ph-H); 6.724 (s, 1H, -Ph-H); 6.630 (d, 1H, -Ph-H); 6.335 (s, 1H, -Ph-H); 2.613 (t, 3H, -CH3); TG analysis: residue 19.65% (calculated 18.77%, CoO). Molar conductivity, Λm (S·cm^2^·mol^-1^): 16.91.

C4: yield, 85%; Anal. Calc. for C4 {%, [Co (C_15_H_11_O_2_N_2_) (CH_3_COO)], FW=369.24 g·mol-1}; C, 55.30; H, 3.82; N, 7.59. Found (%): C, 55.01; H, 3.79; N, 7.20. λmax (nm): 237, 286. IR data (KBr, cm^-1^): 3289.67, υ (-NH-); 1672.52, υ (-C=O); 1612.31, υ (-C=N-); 1526.21 υ_as_ (COO-); 1320.54, υ_s_ (COO-); 1226.34, υ (-Ph-OH); 473.04, υ (Co-O). 1H NMR (DMSO, 600 MHz; s, singlet; d, doublet; t, triplet): δ (ppm) 10.496 (s, 1H, -NH-); 7.497 (s, 1H, -Ph-H); 7.340 (d, 1H, -Ph-H); 7.066 (s, 1H, -Ph-H); 6.726 (s, 1H, -Ph-H); 6.462 (s, 1H, -Ph-H); 6.438 (d, 1H, -Ph-H); 6.306 (s, 1H, -Ph-H); 2.614 (t, 3H, -CH3); 2.541 (d, 3H, -CH3). TG analysis: residue 20.95% (calculated 20.29%, CoO). Molar conductivity, Λm (S·cm^2^·mol^-1^): 18.12.

C5: yield, 80%; Anal. Calc. for C5 {%, [Zn (C_19_H_14_O_3_N_3_) (CH_3_COO)], FW=456.77 g·mol^-1^}; C, 55.22; H, 3.75; N, 9.20. Found (%): C, 55.15; H, 3.71; N, 9.52. λmax (nm): 231, 296. IR data (KBr, cm^-1^): 3399.68, υ (-NH-); 1711.36, υ (-C=O); 1611.65, υ (-C=N-); 1608.21, υ_as_ (COO-); 1316.82, υ_s_ (COO-); 452.54, υ (Zn-O). 1H NMR (DMSO, 600 MHz; s, singlet; d, doublet; t, triplet; m, multiplet): δ (ppm) 10.749 (s, 1H, -NH-); 9.762 (s, 1H, -NH-); 7.919 (m, 4H, -Ph-H); 7.497 (s, 1H, -Ph-H); 7.340 (d, 1H, -Ph-H); 7.067 (s, 1H, -Ph-H); 6.724 (s, 1H, -Ph-H); 3.779 (s, 1H, -C-H-); 3.16 (d, 1H, -C-H-); 3.021 (t, 2H, -CH2-); 2.613 (t, 3H, -CH3). TG analysis: residue 19.06% (calculated 18.21%, ZnO). Molar conductivity, Λm (S·cm^2^·mol^-1^): 23.56.

C6: yield, 85%; Anal. Calc. for C6 {%, [Zn (C_17_H_13_O_3_N_2_) (CH_3_COO)], FW=417.73 g·mol-1}; C, 54.63; H, 3.86; N, 6.71. Found (%): C, 54.51; H, 3.81; N, 7.01. λmax (nm): 232, 652. IR data (KBr, cm^-1^): 3267.68, υ (-NH-); 1686.32, υ (-C=O); 1612.55, υ (-C=N-); 1590.95, υ_as_ (COO-); 1339.93, υ_s_ (COO-); 445.30, υ (Zn-O). 1H NMR (DMSO, 600 MHz; s, singlet; d, doublet; t, triplet): δ (ppm) 10.760 (1H, s, -NH-); 7.498 (s, 1H, -Ph-H); 7.342 (d, 1H, -Ph-H); 7.140 (t, 2H, -Ph-H); 7.067 (s, 1H, -Ph-H); 7.050 (t, 2H, -Ph-H); 7.024 (s, 1H, -Ph-H); 6.724 (s, 1H, -Ph-H); 3.779 (s, 1H, -C-H-); 3.020 (t, 2H, -CH2-); 2.614 (t, 3H, -CH3). TG analysis: residue 19.65% (calculated 19.30%, ZnO). Molar conductivity, Λm (S·cm^2^·mol^-1^): 21.42.

### Elemental analysis and NMR spectroscopy

Elemental analysis (C, H and N) was performed using a 2400 PerkinElmer analyzer (Perkin-Elmer, Inc., Wellesley, MA, USA). Infrared spectrum was recorded as KBr pellets on the Nicolet 170SX spectrophotometer (Thermo Fisher Scientific Inc., Waltham, MA, USA) in the 4,000–400 cm^-1^ region. 1H NMR spectrum was recorded on an Avance III (600 MHz) spectrometer (Bruker Biospin Group, Zurich, Switzerland).

### Cell culture and whole-cell extract preparation

MDA-MB-231, LNCaP and PC-3 cell lines were obtained from the American Type Culture Collection (ATCC; Manassas, VA, USA). The MDA-MB-231 human breast cancer cells were cultured in DMEM/F-12 (1:1) and LNCaP and the PC-3 human prostate cancer cells were cultured in RPMI-1640 medium. All media were supplemented with 10% FBS, 100 μg/ml streptomycin and 100 U/ml penicillin (Life Technologies, Carlsbad, CA USA). All cells were maintained in a humidified atmosphere containing 5% CO_2_ at 37°C. The cells were harvested, washed with phosphate-buffered saline (PBS), lysed in lysis buffer [50 mM tris(hydroxymethyl)aminomethane Tris-HCl, pH 8.0, 150 mM NaCl, 0.5% NP40], vortexed at 4°C for 30 min, and centrifuged at 13,000 × g for 14 min (27). The supernatants were collected as whole-cell extracts and used for the measurement of chymotrypsin-like activity and western blot analysis, as previously described (28).

### Cell proliferation assays

The effects of the complexes the growth of cancer cells were determined by MTT assay. The MDA-MB-231 (breast cancer), and the LNCaP and PC-3 (prostate cancer) cells were seeded in triplicate in 96-well plates and cultured until 70–80% confluency at 37°C, followed by treatment with the indicated concentrations of each compound for 24 h. The medium was then removed and MTT solution (1 mg/ml) was added. After 2 h of incubation at 37°C, MTT was removed, and 100 μl DMSO were added to dissolve the metabolized MTT product. The inhibition of cell proliferation was measured at an absorbance of 560 nm on a Wallac Victor3 multi-label plate reader (Perkin-Elmer, Inc.).

### Proteasomal chymotrypsin-like activity in MDA-MB-231 breast cancer cells

The MDA-MB-231 cells were treated with C1-C6 at the indicated concentrations (5, 10, 20, 30, 40 μM) or for different periods of time (0, 2, 4, 8, 16, 24 h; C=30 μM), lysed, and the protein concentrations were measured using a Bio-Rad protein assay (Bio-Rad). Whole-cell lysates (10 μg) were incubated for 2 h at 37°C in 100 μl assay buffer (20 mM Tris-HCl, pH 7.5) with 20 μM fluorogenic peptide substrate Suc-LLVY-AMC (AnaSpec, Fremont, CA, USA). Proteasomal CT-like activity was measured using the Wallac Victor3 multi-label counter with an excitation filter of 365 nm and an emission filter of 460 nm, as previously described (3).

### In vitro proteasomal activity assay in MDA-MB-231 breast cancer cell extracts

The MDA-MB-231 cell extracts (10 μg total protein) were incubated in 100 μl assay buffer (20 mM Tris-HCl, pH 7.5) and 20 μM chymotrypsin-like substrate Suc-LLVY-AMC, with various concentrations of C1-C6 or DMSO as the vehicle control for 2 h at 37°C. Following incubation, proteasome CT-like activity was measured using the Wallac Victor3 multi-label counter with an excitation filter of 365 nm and an emission filter of 460 nm, as previously described (3).

### Western blot analysis

Proteins (30 μg) from whole-cell lysates were separated by sodium dodecyl sulfate polyacrylamide gel electrophoresis (SDS-PAGE) and then transferred onto nitrocellulose membranes. Western blot analysis was performed using specific antibodies against Ub, Bax, PARP and β-actin, followed by visualization with enhanced chemiluminescence reagent (Denville Scientific, Inc., Metuchen, NJ, USA), as previously described (29).

### Analysis of cellular morphology

Cellular morphological changes were observed using an Axiovert 25 phase contrast microscope (Carl Zeiss Inc., Thornwood, NY, USA), as previously described (29).

## Results

### IR spectral studies

The structural explanation of the complexes is supported by infrared spectroscopy (IR spectra). There are medium strong bands at 3,189–3,399 cm^-1^ in the spectra of compounds C1-C6 which are assigned to υ (-NH-) vibration. The IR spectra also shows sharp bands at 1,622–1,636 cm^-1^ corresponding to υ (-C=N-) in ligands that are not shown in this article, which shifted to 1,602–1,618 cm^-1^ in compounds 1-C6, indicating the coordination complex between nitrogen and metal. Further evidence of the complexation of nitrogen is obtained from the appearance of new bands at 445–478 cm^-1^ which is assignable to υ (M–N) for the complexes. The loss of OH proton is indicated by the absence of bands at ~3,500 cm^-1^ in the complexes C1-C6. The difference between the value of υ_as_ (COO-) and υ_s_ (COO-) is greater than 200 cm^-1^, thus confirming that carboxylic radical is in the form of monodentate in the coordination complex.

### Growth inhibitory effect of compounds C1-C6 in MDA-MB-231 breast cancer cells

First, to investigate whether compounds C1-C6 had anti-proliferative ability, the MDA-MB-231 breast cancer cells were treated with 5, 15 or 30 μM of C1 to C6 for 24 h, followed by analysis by MTT assay. Cells treated with DMSO were used as a control. C3 and C5 had similar growth-inhibitory activities, resulting in approximately 50% inhibition at 5 μM, 90 and 82% inhibition at 15 μM, respectively and at >92% inhibition at 30 μM (Fig. 1). C1 was also a potent inhibitor, displaying 5, 12 and 99% in inhibition at 5, 15 and 30 μM, respectively (Fig. 1). However, C2, C4 and C6 showed a slight inhibitory effect at 5, 15, 30 μM after 24 h of treatment (Fig. 1).

### Inhibition of intact 26S proteasome activity by C1-C6 in vitro

To investigate whether these complexes were capable of inhibiting proteasome activity with effects similar to those observed on cell proliferation, the MDA-MB-231 cell extracts were treated with various concentrations of C1-C6 (5, 15, 30 μM) for 2 h, with DMSO treatment as a control, followed by the measurement of proteasomal CT-like activity (using a fluorogenic substrate specific for the CT-like subunit). The results clearly indicated that the compounds C1, C3 and C5 were the most potent against proteasomal chymotrypsin-like activity (Fig. 2), similar to their effects on cell proliferation, while C2, C4 and C6 were much less potent (Fig. 2), similar to their effects on cell proliferation as measured by MTT assay.

### Concentration-dependent proteasome inhibition and induction of apoptosis by C1, but not C2 in MDA-MB-231 cells

To determine whether chemical structure is important for these compounds to inhibit tumor cellular proteasome activity and induce apoptosis, the MDA-MB-231 cells were treated with various concentrations of the cadmium-based compounds, C1 and C2, which are similar in structure, or DMSO as a control, for 24 h. C1 inhibited proteasomal chymotrypsin-like activity in a concentration-dependent manner, inhibiting >90% activity at 40 μM, while C2 showed no inhibitory effect even at 40 μM (Fig. 3A).

The accumulation of target proteins has been shown to be associated with the inhibition of proteasome activity (29). Western blot analysis revealed a dose-dependent accumulation of ubiquitinated proteins induced by treatment with C1 (Fig. 3B).

It has been reported that the inhibition of tumor cellular proteasome activity is also associated with the induction of apoptosis. In the same experiment, apoptosis associated with changes in cellular morphology were also observed in the cells treated with C1 at concentrations as low as 10 μM. These changes did not occur in the cells treated with C2, even at the highest concentration (40 μM) (Fig. 3C). These results suggested that C1, but not C2, inhibited cellular proteasome activity and induced apoptosis in the intact MDA-MB-231 cells.

### Time-dependent proteasome inhibition and induction of cell death by C1, but not C2 in MDA-MB-231 cells

To verify that the observed apoptotic changes were a result of proteasome inhibition, the MDA-MB-231 cells were treated with 30 μM C1 for 0, 2, 4, 8, 16 and 24 h. Treatment with C2 for 24 h served as a control. The results revealed that proteasomal chymotrypsin-like activity was inhibited by 36% in these breast cancer cells after only 2 h of treatment with C1 (Fig. 4A) and further decreased in a time-dependent manner. After 24 h of treatment with C1, proteasomal chymotrypsin-like activity was inhibited by 98%, whereas C2 treatment resulted in only 5% inhibition (Fig. 4A).

Western blot analysis revealed that the accumulation of ubiquitinated proteins appeared at 8 h of treatment with C1 (Fig. 4B). Morphological changes, indicative of cellular apoptosis, were observed after 8 h of treatment with C1 and almost increased to 100% after 24 h (Fig. 4C). By contrast, apoptosis was observed in the cells treated with C2 for 24 h (Fig. 4B and C).

### C3 and C5, but not C4 or C6, has proteasome-inhibitory and apoptosis-inducing activities in MDA-MB-231 cells

To confirm our findings further, we compared the biological activities of another two pairs of complexes [C3 vs. C4 and C5 vs. C6 (Table I)] in the MDA-MB-231 breast cancer cells.

The results indicated that C3 and C5, but not C4 or C6, inhibited the tumor cell proteasome in a dose-dependent manner, as shown by CT-like activity assay (Figs. 5A and 7A). C3 inhibited cell proliferation by 30% at 5 μM and by approximately 50, 75, 81 and 95% at 10, 20, 30 and 40 μM, respectively (Fig. 5A). As shown in Fig. 7A, C5 at 40 μM exhibited marked effects on cellular proteasome activity, causing 96% inhibition. By contrast, C4 and C6 had very little inhibitory effect even at 40 μM (Figs. 5A and 7A). The levels of Bax increased at 20 μM and, more clearly, at 40 μM in the MDA-MB-231 cells treated with C3 (Fig. 5B). They were observed at 5 μM, with the highest levels at 40 μM following treatment with C5 (Fig. 7B). The 85 kDa PARP cleaved fragment appeared at DMSO treatment and accumulated in a dose-dependent manner, while it appeared at 5 μM C5 treatment and accumulated as the C5 dose increased (Figs. 5B and 7B). However, slight accumulation was observed when 40 μM of C4 and C6 was used in the MDA-MB-231 cells (Figs. 5B and 7B). The MDA-MB-231 cells began to show morphological signs of apoptosis at 20 μM C3 and C5 treatment, with 100% cell death at 40 μM, whereas almost no morphological changes were observed in the cells treated with C4 and C6 at 40 μM (Figs. 5C and 7C).

A kinetic experiment also indicated that the MDA-MB-231 cells treated with C3 and C5 demonstrated time-dependent proteasome inhibition from 2 to 24 h (Figs. 6A and 8A), which was associated with the accumulation of ubiquitinated proteins, the increased levels of Bax, increased PARP cleavage and increased morphological changes (Figs. 6B and C; 8B and C). On the contrary, treatment with C4 and C6 for 24 h failed to generate any of the above effects except for a modest decrease in CT-like activity (Figs. 6 and 8).

## Discussion

We have previously reported that metal-based proteasome inhibitors potently induce apoptosis (30,31). However, the structure-activity relationship between the metal-based complexes and mechanisms of inhibition remains undefined. One overarching hypothesis in our study is that the structure of the complexes affects the delivery of the metal to the proteasome, causing proteasome inhibition through direct interaction and tumor cell death. In order to investigate whether specific structures have the structure-activity relationship, we synthesized six novel Schiff base complexes that contained different metals and tested their biological activity.

First, we measured the anti-proliferative activity of these complexes by MTT assay (Fig. 1) and found that C1, C3 and C5 possessed a strong ability to inhibit cell proliferation in breast cancer cells in a concentration-dependent manner, whereas C2, C4 and C6 did not. In addition, C1, C3 and C5 at 30 μM inhibited the proliferation of the MDA-MB-231 cells by 99, 95 and 90%, respectively, after 24 h of treatment (Fig. 1). Secondly, we investigated whether these compounds were capable of proteasome inhibition using MDA-MB-231 breast cancer cell extracts (Fig. 2). C1, C3 and C5 inhibited the proteasomal CT-like activity (Fig. 2), and proteasome inhibition was confirmed by the increased levels of the proteasome target protein, Bax, as shown by western blot analysis, in dose- and time-dependent experiments. By contrast, C2, C4 and C6 had little to no proteasome-inhibitory and cell death-inducing activities in the MDA-MB-231 cells.

In this study, we compared the structures and proteasome-inhibitory potential of various metal-containing complexes (Figs. 1 and 2; Table I). While C2 has a very similar structure to C1, their activities differ greatly (Figs. 3 and 4). The structural difference between C1 and C2 is that C1 has a functional methoxyl group, while C2 has only a methyl group. It is well established that the CT-like activity of the 26S proteasome, which is primarily associated with the β5 subunit, depends on the presence of the N-terminal threonine residue that is responsible for catalyzing the cleavage of peptides by nucleophilic attack (32). It is also known that methoxyl attracts with electron groups which easily occurs during nucleophilic attack, particularly with aromatic compounds (33,34). Thus, we hypothesized that the aromatic compounds with electron-attracting cabailities, such as methoxyl, can change the electron density and make metal complexes highly susceptible to nucleophilic attack and therefore likely to inhibit proteasomal CT-like function.

In order to test the aforementioned hypothesis, we investigated the structure and activity of three paired complexes, i.e., C2-C4, C3-C4 and C5-C6 (Figs. 1–8 and Table I). The result indicated that the compounds C2 and C4 had almost the same structure, but not the same metal base. We changed the metal and found that there was no change in the activity (Figs. 3–6). Additionally, we found that the cobalt-based C3 complex had very a similar structure to, but more activity than C4 (Figs. 5 and 6). This inhibitory activity was strongly associated with the abrogation (>90% at 40 μM) of the CT-like activity of the proteasome (Fig. 5A), the accumulation of ubiquitinated proteins, and the aggregation of a prime proteasome target protein, Bax (Figs. 5B and 6B), indicating the occurrence of apoptosis, which was also associated with phenotypic morphological changes (Figs. 5C and 7C). This may be due to the fact that C3 has the electron-attracting carboxyl group, whereas C4 does not (Table I). Similar results were observed in the cobalt-based complexes C5 and C6 (Figs. 7 and 8). The only difference between C5 and C6 was that C5 had an indole ring that is able to attract electron groups.

To confirm our hypothesis further, we investigated the effect of each complex in human prostate cancer cells (LNCaP and PC-3 cells) with the same concentration treatments. The results showed that the complexes C1, C3 and C5 were potent inhibitors of cell proliferation. These results were similar to those observed in the MDA-MB-231 breast cancer cells (data not shown).

All the experiments showed that C1, C3 and C5 had inhibitory activity. The preliminary mechanism of the activity is possibly the special structure, the aromatic ring with electron-attracting cabailities, can transport metal into cancer cells more easily by changing the electron density and nucleophilic attack.

We investigated the growth-inhibitory activity of six metal-based complexes along with their simple mechanism of action. C1, C3 and C5 are potent proteasome inhibitors and apoptosis inducers in some human cancer cells. In conclusion, our study suggests that the metal-based complexes, including aromatic compounds with electron-attracting groups, may be promising in the development of novel anti-cancer drugs.

## Figures and Tables

**Figure 1:** 3-(4,5-Dimethylthiazol-2-yl)-2, 5-diphenyltetrazolium bromide (MTT) assay of metal-based complexes in MDA-MB-231 human breast cancer cells treated with C1-C6. After 24 h, the medium was removed, and the cells were treated with MTT solution, as described in ‘Cell proliferation assays’.

**Figure 2:** CT-activity assay in metal-based complexes in human breast cancer cell (MDA-MB-231) extracts. Total proteins (10 μg) were incubated with various concentrations of C1-C6 for 2 h, followed by proteasomal chymotrypsin-like activity assay. Dimethyl sulfoxide (DMSO) was used as a control.

**Figure 3:** Dose response experiment using C1 and C2 in human breast cancer metal-based complexes in human breast (MDA-MB-231) cells. MDA-MB-231 ells were treated with either solvent dimethyl sulfoxide (DMSO) or C1 and C2 at the indicated concentrations for 24 h. (A) The inhibition of CT-like activity in MDA-MB-231 cells treated with C1 and C2. (B) Western blot analysis using antibodies against ubiquitin (Ub) and β-actin (as a loading control) (C) Cellular morphological changes visualized by phase contrast imaging.

**Figure 4:** Time response experiment using C1 and C2 in human breast cancer metal-based complexes in human breast (MDA-MB-231) cells. MDA-MB-231 cells were treated with 30 μM of C1 and C2 for the indicated times. (A) The inhibition of CT-like activity. (B) Western blot analysis using antibodies to ubiquitin (Ub) and β-actin (as a loading control). (C) Cellular morphological changes visualized by phase contrast imaging.

**Figure 5:** Dose response experiment using C3 and C4 in human breast cancer metal-based complexes in human breast (MDA-MB-231) cells.MDA-MB-231 cells were treated with either solvent dimethyl sulfoxide (DMSO) or C3 and C4 at the indicated concentrations for 24 h. (A) The inhibition of CT-like activity in MDA-MB-231 cells treated with C3 and C4. (B) Western blot analysis using antibodies to proteasome target proteins (Bax), ubiquitin (Ub), poly(ADP-ribose) polymerase (PARP) and β-actin (as a loading control). (C) Cellular morphological changes visualized by phase contrast imaging.

**Figure 6:** Time response experiment using C3 and C4 in human breast cancer metal-based complexes in human breast (MDA-MB-231) cells. MDA-MB-231 cells were treated with 30 μM of C3 and C4 for the indicated times. (A) The inhibition of CT-like activity. (B) Western blot analysis using antibodies to proteasome target proteins (Bax), ubiquitin (Ub), poly(ADP-ribose) polymerase (PARP) and β-actin (as a loading control). (C) Cellular morphological changes visualized by phase contrast imaging.

**Figure 7:** Dose effects of C5 and C6 in MDA-MB-231 human breast cancer cells. MDA-MB-231 cells were treated with either solvent dimethyl sulfoxide (DMSO) or C5 and C6 at the indicated concentrations for 24 h. (A) The inhibition of CT-like activity in the MDA-MB-231 cells treated with C5 and C6. (B) Western blot analysis using antibodies to proteasome target proteins (Bax), ubiquitin (Ub), poly(ADP-ribose) polymerase (PARP) and β-actin (as a loading control) (C) Cellular morphological changes visualized by phase contrast imaging.

**Figure 8:** Tim-response experiment using C5 and C6 in human breast cancer metal-based complexes in human breast cancer (MDA-MB-231) cells. The MDA-MB-231 cells were treated with 30 μM of C5 and C6 for the indicated times. (A) The inhibition of CT-like activity. (B) Western blot analysis using antibodies to proteasome target proteins (Bax), ubiquitin (Ub), poly(ADP-ribose) polymerase (PARP and β-actin (as a loading control). (C) Cellular morphological changes visualized by phase contrast imaging.

**Table I:** Chemical structures of L, N1-N5 and compounds C1-C6.
